The article "The Analysis of How Apnea Influences the Autonomic Nervous System Using Short-Term Heart Rate Variability Indices" was published in 2020. Journal: J Healthc Eng.

# The Analysis of How Apnea Influences the Autonomic Nervous System Using Short-Term Heart Rate Variability Indices

**DOI:** 10.1155/2020/6503715

**Published:** 2020-12-18

**Authors:** Baolin He, Wenyu Li, Xiaotong Zhang, Yanan Wu, Jing Liu, Lara M. Brewer, Lu Yu

**Affiliations:** ^1^Department of Biomedical Engineering, School of Fundamental Sciences, China Medical University, Shenyang, Liaoning, China; ^2^Department of Nuclear Medicine, Zhongnan Hospital of Wuhan University, Wuhan, Hubei, China; ^3^Department of Anesthesiology, University of Utah, Salt Lake, UT, USA

## Abstract

**Objective:**

Frequent cessations of respiration can greatly increase the prevalence rate of arrhythmia. It has been confirmed that cardiac modulation is regulated by the autonomic nervous system (ANS). And heart rate variability (HRV) is widely used as a method to evaluate the function of the ANS. Therefore, we analyzed whether apnea can affect the balance and normal function of the ANS using short-term HRV indices.

**Methods:**

Forty-five healthy subjects were asked to breathe normally and hold their breathing to simulate 10 times apnea. Thirty-six patients from the dataset of a sleep laboratory for the diagnosis of sleep disorders with 10 times apnea were included in analysis. We calculated short-term HRV indices of subjects in normal respiratory and apneic states, respectively.

**Results:**

Compared with the normal respiratory state, respiration cease would lead to the values of Mean-RR, nLF, LF/HF, and *α*1 which significantly increased, whereas the values of rMSSD and nHF significantly decreased.

**Conclusions:**

Cessations of respiration would lead to an imbalance in the function of the ANS, as well as an increase in fractal characteristics of the heart. These changes in the physiological state are likely to induce and cause the occurrence of arrhythmia, which is regulated by the ANS.

## 1. Introduction

People who experience frequent apneic periods initiated by either voluntary or involuntary apnea are more prone to develop cardiac arrhythmia [1]. For example, voluntary breath-holding divers and underwater hockey players are more prone to cardiac arrhythmia [2]. More than 90% of patients with obstructive sleep apnea-hypopnea syndrome, characterized by involuntary apnea during sleep, also have cardiac arrhythmia [3]. The incidence of frequent apneic periods may be a high risk factor for nonorganic cardiac arrhythmia, which is a hallmark of a dysregulated autonomic nervous system (ANS) [4]. We studied whether apneic periods (both voluntary and involuntary apnea) can affect the balance and normal function of the ANS, exhibited by the presence of cardiac arrhythmia. The methods of heart rate variability (HRV), blood pressure monitoring, pulse transit time (PTT), catecholamine assay, and radionuclide imaging [5] can be adopted to evaluate the function of the ANS. Compared with other methods, HRV has the advantages of being noninvasive, quantitative, and simple to calculate. It can analyze the dynamic changes of the ANS more accurately and better evaluate the cardiac sympathovagal balance. We hypothesized that HRV could be used to evaluate the effect of apnea on the function of the ANS.

## 2. Materials and Methods

### 2.1. Subjects

Forty-five healthy male (*n* = 23) and female volunteers (*n* = 22), aged 18–35 years and body mass index (BMI) < 21.4 kg/m^2^, were enrolled in the study after approval for the study protocol was obtained from the Human Institutional Review Board of China Medical University. All subjects gave informed consent before the measurements. They had no extrasystole beats during the measurements. The study was registered at Chinese Clinical Trial Registry (http://www.chictr.org.cn) (ChiCTR-DDD-17014238).

Meanwhile, three hundred subjects were chosen randomly from the dataset of a sleep laboratory for the diagnosis of sleep disorders which is available from PhysioNet (https://physionet.org/physiobank/database/challenge/2018/#files). The subjects had a variety of physiological signals recorded as they slept through the night including electroencephalography (EEG), electrooculography (EOG), electromyography (EMG), electrocardiology (ECG), oxygen saturation (SaO_2_), and nasal flow pressure. Subjects were eligible if they maintained continuous steady breathing for more than 5 minutes and experienced apneic periods (>15 seconds each) more than 10 times during the studied period. The subjects with extrasystole beats were excluded. Thirty-six male (*n* = 11) and female (*n* = 25) subjects, aged 40–82 years, met the eligibility criteria of our study.

### 2.2. Experimental Protocol

We performed two studies to analyze how apnea influences the ANS using HRV indices: study 1 (45 subjects), in which voluntary apnea was used to simulate apnea, and study 2 (36 subjects), in which actual apnea was observed. For studies 1 and 2, absence of the nasal flow pressure signal for more than 15 seconds was considered an apneic event [6].

#### 2.2.1. Study 1

The subjects in the supine position were asked to breathe normally under the resting state for 2 minutes. Then, the subjects were asked to hold their breathing for about 20 seconds to simulate an apneic event. This type of apnea simulation was repeated every 40 seconds for 10 iterations. During the experiment, we used polysomnography (Alice PDx, Amsterdam, Holland) to collect the physiological signals, including ECG and nasal flow pressure. All signals were acquired synchronously via multiple channels. The sampling rate of the ECG and nasal flow pressure signal is 200 Hz.

Nasal flow pressure was used as the reference signal for dividing normal or apneic respiratory events (Figure 1).

HRV analysis was used to evaluate the function of the ANS. In our study, we used R-R intervals of ECG to calculate the HRV indices. We performed wavelet transform [7] on the ECG signal (as shown in Figure 2), which removed the baseline wander, ambient noise, and power line interference in the signal, and highlighted the feature of the *R*-wave. Finally, we identified the *R*-wave using an amplitude threshold. All the *R*-waves were validated and checked manually by visual inspection, despite the robustness of the *R*-wave detection algorithm in a fully automated mode.

In order to explore the changes of the ANS during apnea, HRV indices during the apneic state (20 seconds) were compared with HRV indices during the normal respiratory state (2 minutes). However, some recent research revealed that there were significant differences in certain HRV indices for different lengths of ECG signals [8–10].

In order to effectively and reasonably compare the changes in HRV indices under the normal respiration and apneic states, the ECG signals collected from our pilot experiment were used to screen out the HRV indices which did not change with data length changes. These data were collected while the 44 subjects in study 1 were resting with the supine position for a total of 10 minutes. We separately split the data into 5 minutes, 2 minutes, 40 seconds, and 15 seconds from the initial point of the 10-minute ECG signal and calculated the HRV indices. The four groups of indices were compared with the HRV indices corresponding to the 10-minute data. If there were no significant differences, the index was considered to be available for subsequent analysis.

A total of ten classic HRV indices were calculated [11]. The time domain indices include the following.

Mean-RR (mean of successive normal R-R intervals): it reflects the mean of all R-R intervals, in unit of ms. It can be calculated as

(1) $$\begin{array}{c} \text{mean}=\bar{\text{RR}}=\sum_{i=1}^{N}\left(\frac{{\text{RR}}_{i}}{N}\right). \end{array}$$

SDNN (standard deviation of successive normal R-R intervals): it reflects the magnitude of sympathetic and parasympathetic tone, in unit of ms. It can be calculated as

(2) $$\begin{array}{c} \text{SDNN}=\sqrt{\frac{1}{N}\sum_{i=1}^{N}{\left({\text{RR}}_{i}-\bar{\text{RR}}\right)}^{2}}. \end{array}$$

pNN50 (percentage of difference between adjacent successive normal R-R intervals that are greater than 50 ms): it represents the changes of R-R intervals and reflects vagal modulation, in unit of %. It can be calculated as

(3) $$\begin{array}{c} p\text{NN}50=\left(\frac{\text{NN}50}{\text{TotalNN}}\right)\times 100\%. \end{array}$$

*r*MSSD (square root of the mean squared differences of successive normal R-R intervals): it reflects the vagal parasympathetic modulation, in unit of ms. It can be calculated as

(4) $$\begin{array}{c} \text{rMSSD}=\sqrt{\frac{1}{N-1}\sum_{i=1}^{N-1}{\left(RR_{i+1}-RR_{i}\right)}^{2}}. \end{array}$$

The frequency domain indices calculated with the method of Lomb–Scargle [12] include the following.

The value of nHF (normalized units of the power in the low-frequency band ranging from 0.04 to 0.15 Hz) can reflect vagal modulation. nLF (normalized units of the power in the high-frequency band ranging from 0.15 to 0.4 Hz) is an indicator of sympathetic modulation, and its value can relate to the combination of sympathetic and parasympathetic function. LF/HF (the ratio of the power of LF and HF) is a sensitive indicator of the shift of sympathovagal balance [13]. In our study, the windowed Lomb–Scargle method, which had the window width set at 15 seconds with an overlap of 5 seconds, was used to calculate the power spectral distribution.

Nonlinear domain indices include SD1, SD2, and *α*1. Among them, SD1 and SD2 are obtained based on the method of Poincare plot. SD1 (SD of ellipse width) can reflect the changes of adjacent RR intervals. SD2 (SD of ellipse length) is an indicator to measure the length of Poincare plot, which can reflect the changes of all RR intervals [14]. The fractal scaling exponent *α*1 calculated by detrended fluctuation analysis (DFA) can not only reflect the sympathovagal modulation but also the strength of the fractal characteristics of the heart. It is often used as an indicator to predict the occurrence of heart disease [15].

The screening results of HRV indices are shown in Table 1. We observed that the values of indices decrease significantly with the decrease of data length (*P* < 0.05), such as SDNN, pNN50, SD1, and SD2, but different data lengths have no significant effects on the values of Mean-RR, rMSSD, nLF, nHF, LF/HF, and *α*1 (*P* > 0.05).

Therefore, we calculated and compared the six HRV indices of 45 subjects in the states of normal respiration (2 minutes) and voluntary apnea (20 seconds) to evaluate the effects on the ANS during voluntary apnea, respectively. These six HRV indices were also used in study 2.

#### 2.2.2. Study 2

For the enrolled thirty-six subjects, we selected the 5-minute periods when the subjects maintained the normal breathing state and the periods when apnea appeared 10 times during the sampling period. The ECG and nasal flow pressure signals during these periods were used for subsequent analysis. Nasal flow pressure signal was used as the reference signal to divide the samples into different respiratory states: normal or apneic.

HRV analysis is the method we adopt to evaluate the function of the ANS. In study 2, we also used R-R intervals of ECG to calculate HRV indices. The R-R intervals were determined in the same way as in study 1.

Just like in study 1, we calculated and compared the six HRV indices of the 36 subjects in normal respiratory (5 minutes) and apneic states (>15 seconds) to evaluate its influence on the balance and normal function of the ANS during apnea, respectively.

In studies 1 and 2, the analysis and processing of the signals were performed using MATLAB (version 8.3, Natick, Massachusetts, USA) software.

### 2.3. Statistical Analysis

When HRV indices were screened in study 1, we used the method of paired-sample *t*-tests to compare the HRV indices for 5 minutes, 2 minutes, 40 seconds, and 15 seconds to the HRV indices for 10 minutes. We used the method of paired-sample *t*-tests to compare the six HRV indices under the normal respiratory state (5 minutes) to the indices in the apneic state (>15 seconds). All data were calculated by SPSS (version 22.0, Inc., Chicago, IL, USA) software, and they were presented in the form of mean ± SE. At the same time, *P*=0.05 was defined. When *P* < 0.05, the two groups of data had statistically significant difference. When *P* > 0.05, there was no statistically significant difference between the two groups.

## 3. Results

The results of studies 1 and 2 show that when apnea (either type) occurred, the values of Mean-RR, nLF, LF/HF, and *α*1 increased, and the values of rMSSD and nHF decreased. The HRV indices under different respiratory states in study 1 are shown in Table 2 and Figure 3. Table 2 and Figure 3 show that, for the subjects in study 1, comparing with the normal respiratory state, under the state of voluntary apnea, the value of Mean-RR (10 events of voluntary apnea) is much more significantly increased, and the values of nLF, LF/HF, and *α*1 are significantly increased (≥7 events of voluntary apnea), whereas the value of rMSSD is significantly decreased (10 events of voluntary apnea), and the value of nHF is significantly decreased (8 events of voluntary apnea). For studies 1 and 2, most of *R*-wave points can be detected using the detection algorithm automatically. Less than one percent of the points was corrected manually.

The HRV indices in different respiratory states in study 2 are shown in Table 3 and Figure 4. Table 3 and Figure 4 show that, for the subjects of study 2, comparing with the normal respiratory state, under the apneic state, the values of LF/HF and *α*1 are significantly increased (10 events of apnea), and the values of Mean-RR and nLF are significantly increased (8 events of apnea), whereas the value of rMSSD is significantly decreased (10 events of apnea), and the value of nHF is significantly decreased (8 events of apnea).

The age of the subjects in study 1 was different from that in study 2. By comparing the HRV index values of Tables 2 and 3, we found that the age had an effect on the HRV and ANS. We also found the difference of HRV indices between the male and female subjects. The Mean-RR, rMSSD, nLF, LF/HF, and *α*1 values of female subjects were lower than those of male subjects, and the nHF value of female subjects was higher than that of male subjects. Although gender affected the value of HRV indices, it did not affect the trend of HRV index variation during apnea.

In Tables 2 and 3, few of apnea events led to HRV index changes with no statistical significance, whereas the vast majority of apnea events led to the significant changes in HRV indices statistically. Hence, considering the physiological significance of these HRV indices, we concluded that compared with normal respiration, any form of apnea (simulated or actual apnea) could result in a significant increase in the body's sympathetic modulation and vagal modulation and a significant change in the balance of the ANS, and it also led to an increase in fractal characteristics of the heart.

## 4. Discussion

In this study, the method of short-term HRV was used to measure and evaluate the function of the ANS in normal respiration and apneic states of two groups of subjects. The results showed that compared with the normal respiratory state, simulated apnea (voluntary apnea) and actual apnea (sleep disorder) both lead to a significant increase in the values of Mean-RR, nLF, LF/HF, and *α*1, whereas the values of both rMSSD and nHF significantly decreased, indicating that sympathetic modulation and vagal modulation were significantly enhanced, the balance of the ANS produced significant changes, and the fractal characteristics of the heart were enhanced.

There are many methods for evaluating the function of the ANS, such as PTT, catecholamine assay, blood pressure monitoring, radionuclide imaging, and HRV. Among them, the method of PTT needs to find the *R*-wave of the ECG signal and *P*-wave of the pulse signal to obtain pulse transit time variability (PPTV), which is complicated to implement. The technique of catecholamine assay is capable of qualitatively and quantitatively measuring the function of the ANS. However, the technique of catecholamine assay needs to obtain the content of catecholamine, which is difficult. The method of blood pressure monitoring and radionuclide imaging can only accurately measure sympathetic nerve modulation, but cannot accurately measure vagal modulation. The calculation of HRV is based on the RR interval of the ECG signal. The method of HRV can quantitatively evaluate the function of the ANS. It can not only specifically analyze the changes of sympathetic and parasympathetic nerves but also has the virtues of being noninvasive, simple to calculate, and repeatable [16]. Hence, the method of HRV was chosen to evaluate the function of the ANS in our experiment.

HRV analysis can be performed using different types of indices. Time domain indices can be simply calculated and are intuitive. They have been firstly used in clinical practice, such as Mean-RR and rMSSD. The frequency domain indices can measure sympathovagal modulation; for example, nHF can reflect relative vagal modulation, and nLF can reflect relative sympathetic modulation. Nonlinear domain indices have great advantages in the analysis of the nonstationary signal, which can reflect the characteristics of ECG signal changing over time and the fractal characteristics of the heart, such as *α*1. In our study, time, frequency, and nonlinear domain indices of HRV were used to evaluate the function of the ANS from different angles.

Different studies used different criteria to define apnea. Apnea was defined as a cessation of breath longer than 15 seconds in our study, although the sleep-related breathing disorder studies usually used 10 seconds as the threshold [17]. The criterion for apnea is from our previous studies [6, 18, 19]. We believe that compared with the normal respiratory state, the trend of HRV index variation under the apneic state will not change, although the value of HRV indices might change slightly with different apnea criteria (breath cessation longer or shorter than 15 seconds).

The method of Lomb–Scargle was used when we calculated the frequency domain indices of HRV because the experiments involved the analysis of the short-term ECG signal. This method is based on a least square fit of sinusoids with the calculation performed directly on uneven RR intervals. It does not need to interpolate and resample the original signal, so avoids spectral distortion [20]. Similarly, the method of DFA was chosen when we calculated the nonlinear domain indices because of the short-term ECG signal in our study. The fractal scaling exponent, *α*1, calculated by DFA can accurately analyze ECG, which is a nonstationary signal, and it can better detect the subtle changes of short-term R-R intervals [21].

The reasons for why apnea leads to arrhythmia are multifaceted and complex. From an anatomical point of view, it has been found that the inspiratory muscles are relaxed in the lungs when apnea occurs. Then, the relaxed muscles cause an increase in intrathoracic pressure and hinder the venous return to the right atrium, which reduces the absolute venous pressure. These low-level changes cause the increase of sympathetic modulation through low-pressure baroreceptors, which makes ANS unbalanced and eventually leads to arrhythmia [22]. This study explored the causes of arrhythmia from the changes of ANS function. The experimental results showed that when apnea occurs, increased Mean-RR indicated an increase in vagal modulation, and reduced rMSSD and nHF and increased nLF and LF/HF implied that the human sympathetic modulation was enhanced relatively and the original ANS equilibrium state was broken. Cardiac modulation is regulated by the ANS. When the normal function of the ANS is unbalanced, an abnormal heart rhythm is formed, which induces arrhythmia. Simultaneously enhanced sympathetic and parasympathetic modulations are also the most common trigger in arrhythmia, such as in atrial fibrillations [4]. In addition, some studies have confirmed that the reduction of fractal characteristics of the heart is closely related to the occurrence of cardiac malignant events, such as congestive heart failure [23], whereas the enhancement of fractal characteristics of the heart would cause arrhythmia [24]. Therefore, when apnea occurred, the phenomenon that the value of *α*1 reflecting the strength of the fractal characteristics of the heart was significantly enhanced further explained the process of arrhythmia induced by apnea in this study.

This study had some limitations. Firstly, although the method of short-term HRV can reflect the changes of the ANS during apnea to a certain extent, its accuracy needs to be verified using a more direct method, such as a neural pathway-related approach. Secondly, there is a disagreement regarding the interpretation of nLF as sympathetic modulation, and we have used one of these statements. More research is needed to further confirm whether it can reflect other physiological mechanisms. Thirdly, most of the simulated and actual apnea in our study lasted for only 20 seconds. Our study only revealed how these 20-second apneic periods influence the ANS. The relationship between longer apnea and ANS should be investigated further. Fourthly, for the subjects with extrasystole beats, the influences on the ANS during apnea should be evaluated in the future study.

## 5. Conclusions

We confirm that HRV could be used to evaluate the effect of apnea on the function of the ANS. Our results suggest that both forms of apnea (simulated and actual apnea) result in a significant increase of sympathetic modulation and vagal modulation, leading to an imbalance in the function of the ANS, as well as an increase in fractal characteristics of the heart. These changes in the physiological state are likely to induce and cause the occurrence of arrhythmia. At the same time, we have described algorithms and indices for short-term HRV, which provide a reliable method for future short-term HRV analysis.

## Figures and Tables

**Figure 1:** An example of the subject's nasal flow pressure signal in study 1. The green rectangle represents normal respiratory condition; the red rectangle represents holding simulated apneic event.

**Figure 2:** (a) Original ECG signal (blue). (b) ECG signal after wavelet transform (red).

**Figure 3:** The values of HRV during the normal respiratory condition (dotted line) and voluntary apneic state (bar) in study 1. The values of (a) Mean-RR, (b) rMSSD, (c) nLF, (d) nHF, (e) LF/HF, and (f) *α*1. Values plotted are means ± SE. Statistical significance between the voluntary apneas and normal breathing: ^*∗*^(*P* < 0.05) significant.

**Figure 4:** The values of HRV during the normal respiratory condition (dotted line) and apneic state (bar) in study 2. The values of (a) Mean-RR, (b) rMSSD, (c) nLF, (d) nHF, (e) LF/HF, and (f) *α*1. Values plotted are means ± SE. Statistical significance between the apneas and normal breathing: ^*∗*^(*P* < 0.05) significant.

**Table 1:** Comparison of HRV indices with different data lengths under the normal respiratory condition.

HRV indices	10 min	5 min	2 min	40 s	15 s
Mean-RR (ms)	870.49 ± 19.2	867.16 ± 18.83	864.9 ± 18.89	870.61 ± 21.44	874.51 ± 22
SDNN (ms)	53.34 ± 3.9	50.35 ± 4.1^*∗*^	49.26 ± 4.66	43.82 ± 5.17^*∗*^	41.86 ± 5.44^*∗*^
pNN50 (%)	20.85 ± 2.9	21.22 ± 3	21.05 ± 3.16	17.37 ± 2.95^*∗*^	15.8 ± 3.12^*∗*^
rMSSD (ms)	43.41 ± 3.79	41.59 ± 3.95	41.1 ± 4	40.63 ± 5.17	39.28 ± 5.22
nLF (%)	47.88 ± 2.66	47.95 ± 2.68	50.68 ± 2.92	45.83 ± 3.29	43.79 ± 3.11
nHF (%)	52.12 ± 2.66	52.05 ± 2.68	49.34 ± 2.92	54.17 ± 3.29	56.21 ± 3.11
LF/HF	1.24 ± 0.17	1.32 ± 10.17	1.46 ± 0.19	1.37 ± 0.23	1.13 ± 0.16
SD1	37.7 ± 2.75	35.57 ± 2.89^*∗*^	34.77 ± 3.26	31.06 ± 3.7^*∗*^	26.95 ± 3.57^*∗*^
SD2	65.34 ± 4.79	61.69 ± 5.03^*∗*^	60.37 ± 5.72	53.62 ± 6.3^*∗*^	47.39 ± 6.04^*∗*^
*α*1	0.96 ± 0.03	0.95 ± 0.03	0.97 ± 0.04	0.93 ± 0.05	1.07 ± 0.07

Values are expressed as mean ± SE. Statistical significance between other lengths of the respiratory condition with a length of 10 minutes: ^*∗*^(*P* < 0.05) significant.

**Table 2:** Result of HRV during the normal respiratory condition and voluntary apnea.

	Mean-RR (ms)	rMSSD (ms)	nLF (%)	nHF (%)	LF/HF	*α*1
*Normal*						
Respiratory state	831.59 ± 19.34	41.57 ± 4.62	44.16 ± 2.71	55.84 ± 2.71	1.07 ± 0.15	0.94 ± 0.04
1^st^ voluntary apnea	867.71 ± 22.07^*∗*^	21.16 ± 2.1^*∗*^	52.05 ± 3.29^*∗*^	47.95 ± 3.29^*∗*^	1.79 ± 0.27^*∗*^	1.18 ± 0.09^*∗*^
2^nd^ voluntary apnea	873.36 ± 21.95^*∗*^	20.62 ± 1.83^*∗*^	52.43 ± 2.79^*∗*^	47.57 ± 2.79^*∗*^	1.53 ± 0.21	1.18 ± 0.07^*∗*^
3^rd^ voluntary apnea	874.32 ± 20.98^*∗*^	20.02 ± 1.49^*∗*^	51.96 ± 3.14^*∗*^	48.04 ± 3.14^*∗*^	1.66 ± 0.24^*∗*^	1.05 ± 0.08
4^th^ voluntary apnea	873.23 ± 22.35^*∗*^	21.21 ± 1.64^*∗*^	48.23 ± 3.01	51.77 ± 3.01	1.4 ± 0.23	1.13 ± 0.07^*∗*^
5^th^ voluntary apnea	874.89 ± 21.84^*∗*^	21.45 ± 1.72^*∗*^	52.98 ± 3.51^*∗*^	47.02 ± 3.51^*∗*^	2.1 ± 0.36^*∗*^	1.17 ± 0.07^*∗*^
6^th^ voluntary apnea	874.53 ± 22.33^*∗*^	19.73 ± 1.61^*∗*^	50.73 ± 3.05^*∗*^	49.27 ± 3.05^*∗*^	1.58 ± 0.22^*∗*^	1.21 ± 0.08^*∗*^
7^th^ voluntary apnea	867.8 ± 20.97^*∗*^	21.86 ± 1.98^*∗*^	52.76 ± 3.54^*∗*^	47.24 ± 3.54^*∗*^	2.24 ± 0.43^*∗*^	1.18 ± 0.08^*∗*^
8^th^ voluntary apnea	870.88 ± 20.6^*∗*^	21.17 ± 2.25^*∗*^	49.17 ± 3.16	50.83 ± 3.16	1.5 ± 0.2	1.15 ± 0.09^*∗*^
9^th^ voluntary apnea	871.18 ± 20.56^*∗*^	20.52 ± 1.68^*∗*^	55.91 ± 3.14^*∗*^	44.09 ± 3.14^*∗*^	1.91 ± 0.25^*∗*^	1.35 ± 0.08^*∗*^
10^th^ voluntary apnea	880.8 ± 21.77^*∗*^	21.2 ± 2.08^*∗*^	56 ± 3.11^*∗*^	44 ± 3.11^*∗*^	2 ± 0.25^*∗*^	1.11 ± 0.07

Values are expressed as mean ± SE. Statistical significance between the 10 events of voluntary apnea with normal respiration: ^*∗*^(*P* < 0.05) significant.

**Table 3:** Result of HRV during the normal respiratory condition and apnea.

	Mean-RR (ms)	rMSSD (ms)	nLF (%)	nHF (%)	LF/HF	*α*1
*Normal*						
Respiratory state	928.83 ± 21.99	35.89 ± 4.31	38.22 ± 2.57	61.78 ± 2.57	0.72 ± 0.48	0.82 ± 0.04
1^st^ apnea	966.89 ± 20.89^*∗*^	21.54 ± 2.08^*∗*^	49.09 ± 3.8^*∗*^	50.91 ± 3.8^*∗*^	1.55 ± 0.26^*∗*^	1.22 ± 0.09^*∗*^
2^nd^ apnea	965.96 ± 21.85^*∗*^	20.7 ± 2.39^*∗*^	50.85 ± 3.09^*∗*^	49.15 ± 3.09^*∗*^	1.41 ± 0.18^*∗*^	1.21 ± 0.09^*∗*^
3^rd^ apnea	967.5 ± 23.21^*∗*^	21.19 ± 2.46^*∗*^	48.61 ± 3.39^*∗*^	51.39 ± 3.39^*∗*^	1.51 ± 0.29^*∗*^	1.16 ± 0.09^*∗*^
4^th^ apnea	983.39 ± 22.05^*∗*^	20.23 ± 1.76^*∗*^	48.74 ± 3.22^*∗*^	51.26 ± 3.22^*∗*^	1.25 ± 0.15^*∗*^	1.16 ± 0.09^*∗*^
5^th^ apnea	964.61 ± 20.59^*∗*^	20.42 ± 2.32^*∗*^	44.87 ± 4.2	55.13 ± 4.2	1.48 ± 0.32^*∗*^	1.07 ± 0.1^*∗*^
6^th^ apnea	959.22 ± 21.76	20.55 ± 2.16^*∗*^	51.29 ± 3.35^*∗*^	48.71 ± 3.35^*∗*^	1.54 ± 0.22^*∗*^	1.17 ± 0.08^*∗*^
7^th^ apnea	964.89 ± 21.99^*∗*^	22.36 ± 2.19^*∗*^	46.61 ± 3.51^*∗*^	53.38 ± 3.51^*∗*^	1.35 ± 0.23^*∗*^	1.3 ± 0.11^*∗*^
8^th^ apnea	968.33 ± 21.46^*∗*^	22.22 ± 2.59^*∗*^	44.75 ± 4.23	55.25 ± 4.23	1.42 ± 0.25^*∗*^	1.1 ± 0.09^*∗*^
9^th^ apnea	960.03 ± 22.11	22.61 ± 2.38^*∗*^	50.07 ± 3.3^*∗*^	49.93 ± 3.3^*∗*^	1.49 ± 0.26^*∗*^	1.19 ± 0.1^*∗*^
10^th^ apnea	961.81 ± 20.46^*∗*^	21.79 ± 2.36^*∗*^	45.86 ± 4.03^*∗*^	54.13 ± 4.03^*∗*^	1.6 ± 0.35^*∗*^	1.19 ± 0.1^*∗*^

Values are expressed as mean ± SE. Statistical significance between the 10 events of apnea with normal respiration: ^*∗*^(*P* < 0.05) significant.

## Data Availability

The healthy subject data used to support the findings of this study are available from the corresponding author upon request. The sleep disorder data used to support the findings of this study have been deposited in the PhysioNet repository (https://physionet.org/physiobank/database/challenge/2018/#files).
